# Timosaponin AIII Suppresses RAP1 Signaling Pathway to Enhance the Inhibitory Effect of Paclitaxel on Nasopharyngeal Carcinoma

**DOI:** 10.1155/2022/6756676

**Published:** 2022-05-09

**Authors:** Xiaofeng Li, Wen Lu, Tianjiao Zhou, Feng Zhao, Li Yang

**Affiliations:** ^1^Department of Otorhinolarynology, Head and Neck Surgery, Shanghai Jiao Tong University Affiliated Sixth People's Hospital, Shanghai 200233, China; ^2^Department of Head and Neck Surgery, People's Hospital of Guang'an City, Guang'an 638001, China

## Abstract

Although PTX has been identified as an effective drug for nasopharyngeal carcinoma (NPC) therapy, it has serious side effects in the human body. Previous studies have shown that timosaponin AIII (TSAIII) can inhibit the malignant progression of NPC cells. This study investigated the active mechanism of the combination of TSAIII and paclitaxel (PTX) on NPC. Cellular viability, apoptosis, apoptotic factors, and RAP1 signaling regulators were detected in the PNC cells (CNE-1 and HNE-2) and the subcutaneous CNE-1 transplanted nude mice treated with PTX or/and TSAIII. The results showed that TSAIII notably strengthened the inhibitory effect of PTX on the proliferation of NPC cells CNE-1 and HNE-2; upregulated the expression of Bax B-cell lymphoma 2 (Bcl-2)/Bcl-xL-associated death promoter (Bad), and Ras-associated protein1 (RAP1) GTPase activating protein (Rap1GAP); inhibited the level of Bcl-2, RAP1, and Ras guanine nucleotide releasing protein (RasGRP2); and significantly enhanced the promoting effect of PTX on apoptosis in the CNE-1 and HNE-2 cells. Besides, TSAIII strengthened the inhibitory effect of PTX on xenograft tumor in nude mice without adverse reactions. In conclusion, the combination administration of TSAIII and PTX had a significantly therapeutic effect on NPC and avoided the PTX's side effects, which may have acted as a new direction for the study of therapeutic approaches for NPC clinically.

## 1. Introduction

Nasopharyngeal carcinoma (NPC) is a malignant tumor that occurs in the superior wall (roof) and medial wall of the nasopharyngeal cavity. NPC has an insidious onset and the incidence ranks first among ear, nose, and throat malignancies [1]. Most NPC patients have a more dangerous prognosis due to late diagnosis. So far, radiotherapy is the main treatment manner for NPC. Chemotherapy is regarded as a supplement treatment. However, it is not applicable for patients with advanced NPC because both radiotherapy and chemotherapy can lead to drug tolerance [2]. Despite advanced radiotherapy and chemotherapy techniques now, the 5-year survival rate of the patients with NPC has not been significantly improved yet [3]. Therefore, it is urgent to find a way with high efficacy and less side effects for the treatment of NPC.

Paclitaxel (PTX) belongs to diterpenoid alkaloid compounds, which has been confirmed as the new generation of cancer chemotherapy drug clinically [4]. Clinical studies have confirmed that patients receiving PTX chemotherapy are often prone to various side effects, such as neuropathic pain and myelosuppression [5]. It is reported that drug combination can significantly improve therapeutic efficacy and reduce side effects in the treatment of NPC [6]. Zhou et al. recently showed that some traditional Chinese medicine (TCM) monomers can enhance the antitumor effect of PTX [7]. Hence, the combination of TCM and PTX may be an effective method and reduce side effects for NPC therapy.

Timosaponin AIII (TSAIII), a steroidal saponin, is the main pharmacologically active component in rhizoma anemarrhenae (A Chinese medical herbs) [8]. Some studies have shown that TSAIII has pharmacological effects including anti-inflammation and anticancer [9]. Besides, it is reported that TSAIII not only can significantly promote the apoptosis of melanoma [10], colorectal cancer [11], breast cancer [12], and osteosarcoma [13] but also inhibit their metastatic activity.

Small GTPase Ras-associated protein 1 (RAP1) is a major member of inside-out signaling cascades to activate integrin [14, 15]. Dysfunction of the RAP1 signal involves tumor metastasis and invasion. Activation of the RAP1 signaling is correlated to the aggressive phenotypes of malignancy [16, 17]. Indeed, in the prostate cancer [18], glioblastoma [19], non-small-cell lung cancer [20], melanoma [21], breast cancer [22], and pancreatic cancer [23], RAP1 revealed a prooncogenic activity to promote invasion and migration of tumor cells. On the other hand, GTPase activating protein RAP1GAP acts as a negative regulator of Rap1 activity, which is always found to be downregulated in many cancers [24].

Consequently, this study investigated the effect and the mechanism of the combination of PTX and TSAIII on the occurrence and development of NPC via RAP1 regulation *in vitro* and *in vivo*.

## 2. Materials and Methods

### 2.1. Culture of Cells

Human NPC cell lines CNE-1 and HNE-2 were purchased from Biovector NTCC (Beijing, China). The cells were cultured in RPMI-1640 culture medium with 10% of fetal bovine serum (FBS, Hyclone, Logan, UT, USA) and 1% of penicillin-streptomycin (100 U/mL, Invitrogen; Carlsbad, CA, USA) in an incubator with 5% of CO_2_ at 37°C.

### 2.2. Cellular Viability Assay

The CCK-8 kit (Abcam, Cambridge, United Kingdom) was utilized for the analysis of cellular viability. Firstly, CNE-1 and HNE-2 cells with a density of 5 × 10^3^/mL/well were seeded in a 96-well plate. After adherence of the cells, TSAIII (0, 10, 20, 40, 80, and120 *μ*M) and/or PTX (0, 2, 4, 8, 16, and 32 *μ*M) were/was added in the cells respectively for 72-hour incubation. Subsequently, each well was added 10 *μ*L of CCK-8 reagent for another 4-hour incubation. Then, Synergy HTX Multi-Mode Reader (Agilent Technologies: Richardson, TX) was applied to detect absorbance values of the solutions at 450 nm.

### 2.3. Apoptosis Assay

The cells were treated by TSAIII (10 *μ*M) and/or PTX (8 *μ*M). After 72 h, the cells were digested using trypsin and then collected, washed with precooled PBS, and suspended with 1x binding buffer. Subsequently, the cells were mixed with 5 *μ*L of annexin V-FITC or/and 5 *μ*L of propidium iodide (PI) under a light avoidance condition at ambient temperature for 15 min. After adding 1x binding buffer for the resuspension of the cells, flow cytometry was conducted for the detection of apoptosis.

### 2.4. RT-qPCR

TRIzol reagent (Invitrogen, Carlsbad, CA, USA) was adopted to extract total RNA from the detecting cells. Following, according to the instruction of PrimeScript RT kit (TaKaRa, Tokyo, Japan), mRNA was reverse transcribed into cDNA. The expression of mRNA were determined by RT-qPCR with SYBR green I Master Mix kits (Invitrogen) using corresponding primers (Table 1). In 7500 real-time PCR system (Applied Biosystems, America), GAPDH acted as the internal control.

### 2.5. Experimental Animal

Shanghai Animal Center (Shanghai, China) provided 20 chargeable male BALB/nude mice (age: 4-6 weeks). Shanghai Sixth People's Hospital Affiliated to Shanghai Jiao Tong University approved the animal experiments. And the animal experiments were performed according to the National Institutes of Health Guidelines for Animal Care.

Twenty male BALB/nude mice (age: 4-6 weeks) (Shanghai Animal Center, Shanghai, China) were randomly divided into control, PTX (10 mg/kg), TSAIII (40 mg/kg), and PTX+TSAIII groups (five mice/group). All the mice were injected subcutaneously with 100 *μ*L of phosphate buffer saline (PBS) solution containing 5 × 10^6^ CNE-1 cells in the right axillary region. After four weeks raise, the tumor volume was calculated as 1/2 × (length × width^2^). Four weeks later, the mice were sacrificed. The mice' bodies and the tumor were weighted and recorded. Partial tumor tissues were fixed in 4% of paraformaldehyde for H&E and immunohistochemical staining analyses.

### 2.6. Statistical Analysis

All experiments were independently repeated three times. The statistical analysis of the data was conducted with SPSS 24.0 (IBM-SPSS, Chicago, IL, USA). And the data was presented as mean ± standard deviation (SD). Student's *t*-test and one-way analysis of variance were carried out for the comparisons between two groups and among multiple groups, respectively. The differences were regarded to be significant if *P* < 0.05. All data presentations were plotted with GraphPad Prism 7.0 software (GraphPad Software, San Diego, CA, USA).

## 3. Results

### 3.1. TSAIII Strengthened the Inhibitory Effect of Paclitaxel on the Proliferation of NPC Cells

To examine the effect of TSAIII combined with PTX on NPC development, different concentrations of TSAIII and PTX were utilized to treat CNE-1 and HNE-2 cells *in vitro*. The TSAIII structure was shown in Figure 1(a). Cellular proliferation test revealed that both TSAII and PTX significantly suppressed the cellular proliferation of either HNE-2 or CNE-1 cells in a dose-dependent manner (*P* < 0.05) (Figures 1(b) and 1(c)). Moreover, the inhibitory effect of PTX on the proliferation of CNE-1 and HNE-2 cells was more significant at a concentration of 8 *μ*M (*P* < 0.01) (Figure 1(c)); therefore, the concentration of PTX was determined to be 8 *μ*M in subsequent experiments. Further treatment of the CNE-1 and the HNE-2 cells with both TSAIII and PTX at the same time revealed that the inhibitory effect of the PTX on the cellular proliferation was notably enhanced by TSAIII (*P* < 0.05) (Figure 1(d)) with a dose-dependent manner. These data expressed that TSAII combined with PTX had a synergistic effect on cellular proliferative inhibition in the CNE-1 and the HNE-2 cells.

### 3.2. TSAIII Strengthened the Promoting Effect of PTX on Apoptosis of CNE-1 and HNE-2 cells

To further testify the synergistic effect of TSAIII on the PTX-caused NPC progression, flow cytometry was conducted to detect the cellular apoptosis. The results of the detection indicated that PTX alone significantly promoted cellular apoptosis of CNE-1 and HNE-2 (*P* < 0.05). And the apoptosis was notably higher in the TSAIII+PTX group than that in the PTX or TSAIII alone group (*P* < 0.05) (Figure 2(a)). Western blot detection of the apoptosis-related proteins showed that PTX alone obviously increased Bax and B-cell lymphoma 2 (Bcl-2)/Bcl-xL-associated death promoter (Bad) expression and significantly decreased Bcl-2 expression (*P* < 0.05). Notably, simultaneous supplement with TSAIII strengthened the regulative effect of PTX on the apoptotic proteins. The protein expression of Bax and Bad was further increased, while Bcl-2 expression was further reduced (*P* < 0.05) (Figure 2(b)). These results indicated that TSAIII had a synergistic role in the proapopotic activity of PTX in the CNE-1 and HNE-2 cells.

### 3.3. TSAIII Strengthened the Anti-NPC Effect of PTX by Modulating RAP1 Pathway

The mechanism of the synergistic action of TSAIII and PTX was further investigated. Rap1 is reported to potentially regulate oncogenesis, metastasis, immune evasion, and chemoresistance [24]. RT-qPCR analysis revealed that both PTX and TSAIII could significantly increase the gene expression of *RAP1GAP* and reduce the expression of *RAP1* and *RasGRP2* (*P* < 0.05). Interestingly, the combination of TSAIII and PTX had an enhanced effect on the above gene expression compared with single use of either TSAIII or PTX (*P* < 0.05) (Figures 3(a) and 3(b)), disclosing that the increased inhibitory effect of the combination of TSAIII and PTX on NPC was related to the inhibition of the RAP1 pathway.

### 3.4. TSAIII and PTX Exerted a Synergistic Antitumor Activity In Vivo

A xenograft mouse model was utilized to validate the synergistic antitumor effect of TSAIII and PTX *in vivo*. The results showed that either PTX or TSAIII obviously reduce tumor volume and weight (*P* < 0.05). The inhibitory effect of the combination of PTX with TSAIII on tumor growth was significantly increased (*P* < 0.05) (Figures 4(a)–4(c)). Besides, the weight of the mice in the combined treatment group was not significantly different compared with the control group (*P* > 0.05). These data indicated that combination of PTX with TSAIII had less side effects on the mice (Figure 4(d)). All results above suggested that the synergistic antitumor effect of the combination of TSAIII with PTX was verified as well *in vivo*.

### 3.5. TSAIII Promoted the PTX-Induced Effects on Cellular Apoptosis in Tumor Tissues In Vivo

H&E staining and immunohistochemical assays were processed to determine the cellular apoptosis in the tumor tissues. The H&E staining showed that the apoptotic cells in tumor tissues declined significantly in the TSAIII+PTX group compared with the single administration of either the TSAIII or PTX group (Figure 5(a)). Besides, the immunohistochemical assays also revealed that the combination of TSAIII with PTX further increased the expression of caspase-3 and Bax in tumor tissues compared with the single administration of either TSAIII or PTX (Figures 5(b) and 5(c)). All the *in vivo* experimental results above demonstrated that TSAIII enhanced the induced effects of PTX on cellular apoptosis in tumor tissues.

## 4. Discussion

It's reported that the most widely applied anticancer drug at present is PTX. However, the resistance of the PTX can cause the failure of the treatment for the cancers [25]. Chen et al. have reported that TCM monomers combined with PTX have been applied as an alternative therapy for the tumors and got good results [26]. In this study, we found that TSAIII significantly strengthened the inhibitory effect of PTX on the NPC growth and metastasis via decreasing the cellular proliferation and increasing the cellular apoptosis *in vitro* and *in vivo*. Detail study of the anti- and proapoptotic regulator balance revealed that TSAIII upregulated the expression level of Bax and Bad but declined the expression level of Bcl-2. Usually, the antiapoptotic and proapoptotic protein regulator balance is a critical important to decide whether the cells go through apoptosis. Deregulation of apoptosis is believed to be one of the cancer's hallmarks [27]. Both Bax and Bad are the crucial proapoptotic regulators, while Bcl-2 is an important antiapoptotic factor. All of them are involved in the regulation of extrinsic apoptotic pathway [28]. Thus, TSAIII strengthened the antioncogenesis of PTX on the NPCs through downregulation of Bax and Bad and upregulation of Bcl-2 to improve the NPC apoptosis. We noticed that either PTX or TSAIII alone exhibited the antitumor activity via Bax and Bad inhibition and Bcl-2 elevation to prohibit PNC proliferation and improve apoptosis. Interestingly, the combination of PTX with TSAIII created more effective antitumor activity than single use of either PTX or TSAIII, mechanically, which revealed more inhibitory effect on Bax and Bad, but more activation power on Bcl-2 to much inhibit proliferation and much improver apoptosis in the PNCs. More importantly, combination administration of PTX with TSAIII did not show obvious side effects in the xenograft mouse model assay, because the body weight between the PTX+TSAIII group and either PTX or TSAIII group did not have any significant difference.

RAP1 is a GTPase protein that can interact with other proteins to regulate physiological and pathological processes such as migration, invasion, and metastasis of tumor cells [29–31]. Lost control of the RAP1 signal is associated with tumor growth and metastasis. RAP1 signaling activation is reported in many types of cancers [18–20, 22]. Inactivation form of RAP1 (RAP1-GDP) is positively regulated by guanine nucleotide exchange factors (GEFs), including cAMP, Epac, C3G, RapGRP2, and PDZ-GEF, to form a Rap1-GTP (activation form). On the other hand, the activated form of Rap1-GTP is negatively regulated by GTPase activation proteins (GAPs), including Rap1GAP and SPA-1 [24]. Our data showed that combination of the PTX with TSAIII improved the inhibitory effect of RAP1 and RasGRP2 induced by either PTX or TSAIII alone, further inhibiting the PNC growth. It has been shown that CD38 can promote RasGRP2/RAP1-mediated adhesion and migration of chronic lymphocytic leukemia cells by increasing intracellular Ca^2+^ levels [32]. However, either PTX or TSAIII also revealed the prohibited activity on Rap1-GAP. A study shows Rap1GAP as a tumor suppressor can inhibit the development and progression of many tumors [33, 34]. Therefore, the balance of RasGRP2 and RAP1 with Rap1-GAP will decide the tumor direction. Thus, our results verified that TSAIII inhibited PNC growth via the inhibition of the RAP1 pathway in CNE-1 and HNE-2 cells, thereby playing a synergistic role with PTX to prohibit NPC cells. The combined treatment of TSAIII and PTX further emphasized the proapoptotic effect of PTX via RAP1 pathway suppression in NPC cells.

In summary, it is found in this study that, in vitro and *in vivo*, TSAIII has enhanced the anti-tumor effect of PTX on NPC cells. The combination of TSAIII and PTX offers a new research direction for the clinical treatment of NPC. The limitation of this study is the lack of a systemic examination of the side effect of the PTX+TSAIII combination on the hematological, hepatic, renal, and cardiological systems in the xenograft mouse model.

## Figures and Tables

**Figure 1:** Effect of TSAIII combined with PTX on cellular proliferation of the nasopharyngeal carcinoma cells (PNCs). (a) Chemical structure of TSAIII. (b–d) CCK-8 was applied to test the cell viability of CNE-1 and HNE-2 cells treated by TSAIII (b), PTX (c), and PTX0+TSAIII (d). ^∗^*P* < 0.05 and ^∗∗^*P* < 0.01 vs. the 0.0 *μ*M group, ^##^*P* < 0.01 vs. the 8 *μ*M PTX or 5 *μ*M TSAIII.

**Figure 2:** Effect of combination of TSAIII and PTX on apoptosis of the PNCs. (a) Flow cytometry was utilized to determine the cellular apoptosis in the indicated group of CNE-1 and HNE-2 cells. (b) RT-qPCR was applied to test the mRNA expression of Bax, Bad, and Bcl-2 in CNE-1 and HNE-2 cells. ^∗^*P* < 0.05 and ^∗∗^*P* < 0.01 vs. the control group; ^#^*P* < 0.05 and ^##^*P* < 0.01 vs. 8 *μ*M PTX or 10 *μ*M TSAIII.

**Figure 3:** Effect of combination of TSAII and PTX on RAP1 pathway-regulating factors in the NPCs. RT-qPCR was applied to analyze the mRNA levels of RAP1 pathway-regulating factors in the indicated group of CNE-1 (a) and HNE-2 (b) cells. ^∗∗^*P* < 0.01 vs. the control group; ^##^*P* < 0.01 vs. 8 *μ*M PTX or 10 *μ*M TSAIII.

**Figure 4:** Effect of TSAIII combined with PTX on the growth of transplanted PNC tumor in nude mice. Images showed the tumor size (a), volume (b), weight (c), and nude mice weight (*n* = 5) (d) 4 weeks after inoculation of the xenografts tumor in nude mice at the indicated conditions. ^∗∗^*P* < 0.01 vs. the control group; ^#^*P* < 0.05 vs. 10 mg/kg PTX or 40 mg/kg TSAIII.

**Figure 5:** Effect of TSAIII combined with PTX on cell apoptosis in tumor tissue of the nude mice. (a) H&E staining was utilized to check the cell apoptosis in tumor tissues of the indicated group. Immunohistochemical staining was performed to determine caspase-3 (b) and Bax (c) expressions in the PNC tumor tissues of the indicated group.

**Table 1:** 

Gene	Primer sequence (5′-3′)
Bax	Forward: 5′-CCCGAGAGGTCTTTTTCCGAG-3′
	Reverse: 5′-CCAGCCCATGATGGTTCTGAT-3′
Bad	Forward: 5′-CCCAGAGTTTGAGCCGAGTG-3′
	Reverse: 5′-CCCATCCCTTCGTCGTCCT-3′
Bcl-2	Forward: 5′-CGGTTCAGGTACTCAGTCATCC-3′
	Reverse: 5′-GGTGGGGTCATGTGTGTGG-3′
RAP1	Forward: 5′-GCGAGTAGTTGGCAAAGAGC-3′
	Reverse: 5′-ACTATGGGCCTAGAGCAGCA-3′
RAP1GAP	Forward: 5′-CTACCGGAAGCACTTTCTCG-3′
	Reverse: 5′-CACACACCAACTTTGCCAT-3′
RasGRP2	Forward: 5′-ACAATCCCGGAAGGACAACTC-3′
	Reverse: 5′-GTCTATGTCGATTAGGCTGCTG-3′
GAPDH	Forward: 5′-GCACCGTCAAGGCTGAGAAC-3′
	Reverse: 5′-TGGTGAAGACGCCAGTGGA-3′

## Data Availability

The data used to support the findings of this study are available from the corresponding author upon request.
